The article "The Multiple Pharmacologic Functions and Mechanisms of Action of Guizhi Fuling Formulation" was published in 2022. Journal: Evid Based Complement Alternat Med.

# The Multiple Pharmacologic Functions and Mechanisms of Action of Guizhi Fuling Formulation

**DOI:** 10.1155/2022/6813421

**Published:** 2022-04-29

**Authors:** Jie Gao, Jianmei Yang, Zhiyuan Lu, Xianwen Dong, Ying Xu

**Affiliations:** ^1^Department of Physiology, School of Basic Medicine, Shanghai University of Traditional Chinese Medicine, 1200 Cailun Road, Shanghai 201203, China; ^2^Department of Rehabilitation Medicine, Affiliated Hospital of Nantong University, 20 Xisi Road, Nantong 226001, Jiangsu, China; ^3^Department of Traditional Chinese Medicine, Shanghai Xuhui District Central Hospital, Shanghai 200031, China; ^4^Department of Children Rehabilitation Medicine, The Fifth Affiliated Hospital of Zhengzhou University, Zhengzhou 450052, China

## Abstract

**Objectives:**

Guizhi Fuling Formulation (GZFL), a traditional Chinese medical formulation, consists of Cinnamomi Ramulus, Paeoniae Radix Alba (or Paeoniae Radix Rubra), Moutan Cortex, Persicae Semen, and Poria, with multiple therapeutic functions such as sedation, antitumor activity, anti-inflammation, and neuroprotection. However, its clinical applications remain relatively fragmented, and the underlying mechanisms of GZFL in different diseases are still not very certain. Further research and summary in both application and mechanisms remain to be needed for human health and the best use of GZFL. Therefore, we summarized the multiple pharmacologic effects and possible mechanisms of action of GZFL according to recent 17 years of research.

**Methods:**

We retrieved four English and two Chinese databases using these keywords (the formulation name or its synonyms) and searched articles written in English from January 2006 up to February 2022. *Key Findings*. GZFL exhibits multiple pharmacologic advantages in gynecologic diseases and other expanding diseases such as cancer, blood, and vascular disease, renal failure, inflammation, and brain injury. Possibly due to its diverse bioactive components and pharmacologic activities, GZFL could target the multiple signaling pathways involved in regulating blood circulation, inflammatory and immune factors, proliferation, apoptosis, and so on.

**Conclusion:**

This review suggests that GZFL displays promising therapeutic effects for many kinds of diseases, which have been beyond the scope of the original prescription for gynecologic diseases. In this way, we wish to provide a reference and recommendation for further preclinic and clinic studies.

## 1. Introduction

Guizhi Fuling Formulation (GZFL) is an ancient Chinese herbal formulation. GZFL was recorded first in *Synopsis of Prescriptions of the Golden Chamber* (https://apps.who.int/iris/handle/10665/206952). This classic tome of traditional Chinese medicine was written by Zhang Zhongjing (AD 150–219), a renowned physician of the Eastern Han Dynasty (AD 25–220).

The article "The Multiple Pharmacologic Functions and Mechanisms of Action of Guizhi Fuling Formulation" was published in 2022. Journal: Evid Based Complement Alternat Med.

GZFL is composed of five herbal ingredients according to Chinese Pharmacopeia: Cinnamomi Ramulus (*Cinnamomum cassia* Presl), Paeoniae Radix Alba/Paeoniae Radix Rubra (*Paeonia lactiflora* Pall and *Paeonia veitchii* Lynch), Moutan Cortex (*Paeonia suffruticosa* Andrews), Persicae Semen (*Prunus persica (L*.) Batsch *and Prunus davidiana* (Carr.) Franch), and Poria (*Poria cocos* (Schw.) Wolf) [1]. The five herbal ingredients from GZFL are mixed at the same ratio in preparations including honey pills, capsules, decoctions, and tablets for the therapeutic method of different diseases. In addition, GZFL is termed differently in different countries: “Guizhi Fuling Wan”, “Guizhi Fuling decoction”, “Guizhi Fuling capsule”, and “Guizhi Fuling tablets” in China; Keishibukuryogan (KBG), K-06, and TJ-25 in Japan; Gyejibokryeong-hwan (GBH) in Korean; and TU-025 in the USA [2–4]. GZFL has been used in different countries. However, the scientific botanical species of these five herbal ingredients are different according to Pharmacopeia in different countries. For example, KBG consists of the Cinnamomi cortex, Radix Paeoniae, Cortex Moutan, Poria, and Semen Persicae. GBH is composed of Cinnamomi Ramulus, Poria, Moutan Cortex, Semen Persicae, and Paeoniae radix. TU-025 comprises Cinnamon bark, Peony root, Peach kernel, Poria sclerotium, and Moutan bark.

GZFL was utilized widely to invigorate blood circulation and remove blood stasis. It has achieved obvious effects on various gynecologic diseases in China for more than 1000 years, such as dysmenorrheal, ovarian cysts, and uterine fibroids [5]. Moreover, an increasing number of clinical and experimental data have demonstrated that GZFL possesses potent sedative, analgesic, antitumor, anti-inflammatory, and neuroprotective properties without eliciting adverse effects [6]. Thus, GZFL has also been used to treat microvascular inflammation in the skin [7], bladder cancer [8], uterine fibroids [9], and brain injury [10]. Due to these multiple and attractive therapeutic functions, the bioactivity of GZFL has gained enormous attention, thereby leading to the increasing interest in exploring its pharmacological functions and mechanisms of action.

The active ingredients from GZFL are complex. Pharmacologic studies have shown that GZFL consists of cinnamic acid, cinnamaldehyde, paeoniflorin, albiflorin, gallic acid, ethyl gallate, benzoylpaeoniflorin, and benzoic acid [11–13]. Cinnamic acid and cinnamaldehyde are derived from the crude drugs of Cinnamomi Ramulus, which has antimicrobial, anti-inflammatory, and neuroprotective effects [14–16] and has also been reported to be an immune suppressor [17]. Paeoniflorin and albiflorin are derived from Paeoniae Radix Alba. Paeoniflorin can alleviate some inflammatory and autoimmune diseases, such as endoplasmic reticulum stress-associated vascular inflammation [18] and rheumatoid arthritis [19], and also has improving effects on glutamate-induced damage in PC12 cells and bupivacaine-induced cytotoxicity in SH-SY5Y cells [20, 21]. Albiflorin has antidepressant-like effects by increasing hippocampal expression of 5-hydroxytryptamine (5-HT)/norepinephrine (NE) and brain-derived neurotrophic factor (BDNF) [22] and also ameliorates obesity by modulating the expression of thermogenic genes [23]. Gallic acid and ethyl gallate are derived from Moutan Cortex. Gallic acid can improve ulcerative colitis by suppressing inflammation [24] and also exert neuroprotective effects on memory and long-term potentiation (LTP) impairment by decreasing lipid peroxidation and expression of proinflammatory cytokines in the cortex of rats with traumatic brain injury [25]. Ethyl gallate exhibits antioxidant and anticancer capacities in mice with oral cancer [26]. Benzoylpaeoniflorin and benzoic acids are the main active ingredients of Paeoniae Radix and Moutan Cortex, which can prevent hydrogen peroxide (H_2_O_2_)-induced cytotoxicity in primary neurons from the rat cortex and improve dysmenorrhea by suppressing uterus contraction [27]. However, the synergistic interactions of active ingredients remain unclear and the underlying mechanisms of GZFL in different diseases, such as gynecologic diseases, cancers, blood, and vascular disease, are still not very certain.

The article "The Multiple Pharmacologic Functions and Mechanisms of Action of Guizhi Fuling Formulation" was published in 2022. Journal: Evid Based Complement Alternat Med.

Therefore, in this review, we summarize the clinical therapeutic efficacy and pharmacologic mechanisms of GZFL documented in clinical and experimental studies in recent years, trying to explain the underlying mechanisms in different diseases which may instruct clinical treatment in the future.

## 2. Methods

We retrieved four English and two Chinese databases (PubMed, Web of Science, Science Direct, Wiley Online Library, CNKI, Wanfang Data), combining searching these keywords (the formulation name or its synonyms) in the Medical Subject Headings (MeSH) field and in the title/abstract. All types of clinical and experimental investigations were considered for inclusion. We only searched articles written in English and published in peer-reviewed journals from January 2006 up to February 2022. Studies using GZFL in any preparations (pills, capsules, decoctions, and tablets) were included. The studies which involved the following ineligible interventions were excluded: (1) combined other herbs, modified GZFL, or active ingredients from GZFL; (2) qualitative assessments and studies without statistical significance; (3) GZFL utilized external or topical administration methods. The name of each herbal ingredient was included according to the *Chinese Pharmacopeia*.

The article "The Multiple Pharmacologic Functions and Mechanisms of Action of Guizhi Fuling Formulation" was published in 2022. Journal: Evid Based Complement Alternat Med.

## 3. Gynecologic Diseases

### 3.1. Dysmenorrhea

Dysmenorrhea is the most common gynecologic disorder. It presents as cramps in the abdomen/back during/before menstruation. The main contributor to dysmenorrhea is obviously reduced blood flow caused by enhanced activities and abnormal contractions of the uterus, which induces sensitization of peripheral nerves [28].

A clinical research indicated that GZFL displayed obviously therapeutic effects on patients with primary and secondary dysmenorrhea with the indications such as sweating, heat intolerance, cold sensation in the lower back, and a tense abdomen [29, 30]. GZFL is used widely to treat secondary dysmenorrhea with uterine fibroids. A randomized clinical trial reported that GZFL significantly alleviated dysmenorrhea in patients with uterine fibroids by improving blood stasis and inducing smooth blood flow [3, 4]. In addition, one randomized controlled trial provided support for the positive effects of GZFL on dysmenorrhea and the accompanying acne vulgaris related to menstruation in adults women [12].

Various experimental studies have been carried out to analyze the pharmacologic mechanisms of GZFL in dysmenorrhea. It was reported that GZFL effectively reduced lamina propria edema and displayed a directly inhibitory effect against cyclooxygenase-2 (COX-2) expression, but there is no effect on COX-2 expression in the uterine tissues of oxytocin-induced ICR mice [31]. However, a study in human umbilical vein endothelial cells showed that GZFLs act on downregulating the mRNA levels of COX-1 and COX-2 [32]. Moreover, another *in vivo* study has demonstrated that GZFL significantly improved primary dysmenorrhea with uterine contraction by decreasing the releases of nitric oxide (NO), prostaglandin (PG) F_2a_, Ca^2+^ concentration, expression of COX-2, and oxytocin receptor in the uterine tissue of oxytocin-induced mice. At the same time, GZFL and its components could suppress spontaneous and oxytocin-induced contractions in uterine strips and reduce intracellular Ca^2+^ levels in oxytocin-induced myometrial cells, suggesting that GZFL might exert relaxant effects upon uterine contraction to relieve pain [33]. In addition, an integrative urinary metabolomic study indicated that GZFL treatment reduced the enhanced writhing times and PGF_2a_/PGE_2_ ratio in plasma of rats with primary dysmenorrhea induced by oxytocin injection. Notably, urinary metabolic deviations of those rats were decreased after GZFL treatment, suggesting that GZFL showed therapeutic effects on primary dysmenorrheal by regulating several metabolic pathways [34].

The article "The Multiple Pharmacologic Functions and Mechanisms of Action of Guizhi Fuling Formulation" was published in 2022. Journal: Evid Based Complement Alternat Med.

To further understand for mechanisms and effects of GZFL on primary dysmenorrhea, a pharmacokinetic-pharmacodynamic (PK-PD) model was applied to study the PK processes of several bioactive ingredients from GZFL in plasma: gallic acid, amygdalin, albiflorin, prunasin, and cinnamic acid. Results showed that GZFL significantly decreased the number of spiral arteries and inflammatory cells in uterine tissues of rats with primary dysmenorrhea induced by estradiol benzoate and oxytocin. Moreover, their bioactive ingredients were likely to have key roles in blocking platelet aggregation and thrombosis by increasing the PGE_2_/PGF_2*α*_ ratio and 6-Keto-Prostaglandin F_1*α*_ (6-Keto-PGF_1*α*_)/thromboxane B_2_ (TXB_2_) ratio in plasma of rats with primary dysmenorrhea after GZFL treatment [35].

Therefore, in light of these clinical and experimental studies, we conclude that GZFL possesses the potential for improving primary and secondary dysmenorrhea by regulating the levels of inflammatory factors, intracellular Ca^2+,^ and several metabolic pathways.

### 3.2. Uterine Fibroids

Uterine fibroids (also termed “uterine leiomyomas” or “uterine myomas”) are the most common benign tumor in fertile women. About 50% of uterine fibroids are symptomatic and elicit abdominal pain or extension during menstruation, pressure symptoms, and fertility problems [36]. Surgery is invasive, and hormonal drugs have obvious side effects, so GZFL and several other herbal medicines have been used widely as an alternative treatment for uterine fibroids in China [37, 38]. GZFL was reported to relieve pelvic pain, alleviate the uterine fibroid symptoms and reduce uterine size and fibroids volume in women with symptomatic uterine fibroids [39]. And meta-analyses of clinical trials have indicated that the combined treatment of GZFL and mifepristone might be more advantageous than the use of mifepristone alone for shrinking the volume of fibroids and reducing uterine size. Meanwhile, GZFL plus mifepristone showed less adverse events in comparison to mifepristone alone [3]. Previous research reported that GZFL drug serum was collected from Sprague Dawley (SD) rats and used to treat uterine leiomyoma cells in patients. Results showed that GZFL drug serum possessed the potential to inhibit the proliferation and promote the apoptosis of leiomyoma cells by enhancing the expression of tuberous sclerosis 2 (TSC2) and forkhead box O (FOXO), which are associated with the 14-3-3*γ* signal pathway [40]. However, one study on SD rats model of uterine fibroids and human uterine leiomyoma cells demonstrated that GZFL inhibited uterine fibroids growth by modulating Mediator complex subunit 12 (Med12)-mediated wingless-type (Wnt)/*β*-Catenin signaling pathway [41]. Another research on estradiol-induced endometrial hyperplasia mice showed GZFL ameliorated endometrial hyperplasia through promoting p62-Keap1-NRF2-mediated ferroptosis [42]. The therapeutic mechanism seems multiple. A network pharmacology method was used to identify the pharmacologic mechanism of GZFL against uterine fibroids at the systematic level. This investigation indicated that GZFL exhibited significant therapeutic effects on uterine fibroids through inhibiting proliferation and promoting apoptosis by multiple signaling pathways: Wnt/*β*-catenin, retinoic acid (RA), epidermal growth factor (EGF), and insulin-like growth factor-1 (IGF-1) [9].

The article "The Multiple Pharmacologic Functions and Mechanisms of Action of Guizhi Fuling Formulation" was published in 2022. Journal: Evid Based Complement Alternat Med.

### 3.3. Endometriosis

About 10% of reproductive-age women suffer from endometriosis, a common estrogen-dependent benign disease, which is characterized by pelvic pain, dysmenorrhea, and infertility [43]. In Asia, several herbal formulations (including GZFL) are widely accepted as a kind of alternative medicine to treat endometriosis [44].

Meta-analyses of 10 randomized controlled trials involving 1052 women with endometriosis demonstrated that the combined treatment of GZFL and mifepristone (progesterone antagonist) had obvious benefits in terms of improving the prevalence of pregnancy and decreasing the prevalence of recurrence of endometriosis compared with the use of mifepristone alone. Similarly, GZFL also exhibited adjuvant effects on reducing the level of estradiol and progesterone in the serum of women with endometriosis without serious adverse effects. Thus, GZFL is considered to be an add-on therapeutic approach for endometriosis patients [45].

Furthermore, studies on pharmacologic mechanisms have reported that GZFL can induce serious apoptosis and deter the proliferation and metastasis of endometrial cells in a rat with endometriosis by reversing suppression of survivin and the B-cell lymphoma (Bcl)-2/BCL2-associated *X* protein (Bax) ratio, which is related to the mitochondrial apoptotic pathway. Thus, GZFL is considered to be a potent apoptosis inducer and a therapeutic drug for endometriosis [46].

In addition, GZFL has been shown to significantly lower the volume of endometrial explants in endometriosis rats by immunologic regulation, including decreasing expressions of monocyte chemoattractant protein (MCP)-1 and intercellular adhesion molecules (ICAM)-1 and increasing the number of cluster of differentiation (CD)4^+^ lymphocytes and the activity of natural killer (NK) cells [47].

The article "The Multiple Pharmacologic Functions and Mechanisms of Action of Guizhi Fuling Formulation" was published in 2022. Journal: Evid Based Complement Alternat Med.

In general, the pharmacologic mechanisms of GZFL in improving endometriosis could involve regulating apoptosis and the inflammatory responses as well as other targets.

### 3.4. Climacteric Syndrome

Climacteric syndrome is caused by a decrease in hormonal activity during menopause. This leads to vasomotor symptoms, mood disorders, night sweats, hot flashes, insomnia, and osteoporosis [48–50]. These symptoms usually affect a woman's quality of life severely.

Accumulating studies have shown that the use of herbal medicine is an alternative method for improving climacteric syndrome in women who cannot receive hormone replacement therapy [51, 52]. One clinical study found that GZFL treatment for 12 weeks elicited significant beneficial effects for patients with climacteric symptoms, such as vasomotor symptoms and melancholia. Moreover, the therapeutic effects of GZFL on these patients could be evaluated by identifying a polymorphism of the estrogen receptor *β* (ER*β*) gene, which is involved in climacteric disorders [51]. In perimenopausal and postmenopausal women in Japan, GZFL treatment was shown to be more efficacious than other Kampo formulations in terms of improving sleep disturbance, perspiration, and reducing blood pressure and heart rate [52]. In addition, various studies have shown that GZFL displays beneficial effects on hot flashes in menopausal women [53]. A retrospective case series reported that young women with hot flashes showed improvement after GZFL treatment, possibly by regulating a calcitonin gene-related peptide- (CGRP-) induced temperature rise on the skin without estrogenic activity [54]. Furthermore, a randomized controlled trial in the USA demonstrated that GZFL could obviously decrease the frequency and severity of hot flashes when compared before and after a 3-month intervention in postmenopausal women. However, unlike the clinical experience in Asia, GZFL did not significantly ameliorate hot flashes or sleep quality compared with that obtained using a placebo. This study suggested that future investigations on traditional Asian medicines should consider several potentially important methodological factors [2].

These clinical studies detailed above demonstrated the therapeutic potential of GZFL for the climacteric syndrome.

### 3.5. Polycystic Ovary Syndrome

Polycystic ovary syndrome (PCOS) is a common reproductive endocrine disease in women and the etiology is complex. Besides reproductive dysfunction, the pathological manifestations of PCOS commonly involve insulin resistance and hyperandrogenism [55, 56] and display an inflammatory state [57].

The article "The Multiple Pharmacologic Functions and Mechanisms of Action of Guizhi Fuling Formulation" was published in 2022. Journal: Evid Based Complement Alternat Med.

Studies *in vivo* have reported that GZFL efficiently reduced fasting blood glucose, fasting insulin level, and insulin resistance index in plasma of PCOS rats with insulin resistance [58, 59]. The amelioration of insulin resistance was claimed under the mechanism of regulating intestinal flora to reduce tumor necrosis factor-*α* (TNF-*α*), interleukin-6 (IL-6), and hypersensitive C-reactive protein (HS-CRP) in plasma [58]. In addition, the GZFL-treated rats had lower productions of testosterone, luteinizing hormone (LH), and follicle-stimulating hormone (FSH) compared with PCOS rats and lower LH/FSH ratios. These beneficial tends for normal ovulation were due to the GZFL's effects on inhibiting granulosa cell autophagy and promoting follicular development via restoring the phosphatidylinositol-3-kinase (PI3K)/AKT/mammalian target of rapamycin (mTOR) pathway [59].

## 4. Cancers

### 4.1. Bladder Cancer

Studies have indicated the suppressive effects of GZFL on bladder cancer *in vitro* and *in vivo*. For instance, *in vitro* data indicated that GZFL interfered with cell-cycle progression *via* activation of phosphorylated cell cycle checkpoint kinase2 (CHK2) and cell cycle regulatory protein P21, and induction of apoptosis, in human bladder cancer cell lines. However, GZFL exhibited only weak toxicity to normal human urothelial cells [60]. Another molecular mechanism demonstrates that GZFL could arrest cell cycles efficiently, suppress proliferation, and induce apoptosis in mouse bladder cancer cells (MB49) through increasing levels of reactive oxygen species (ROS) and activating ataxia telangiectasia-mutated (ATM)/CHK2 and ATM/P53 pathways. Furthermore, intravesical GZFL therapy has shown greater inhibitory effects on tumor growth than that of mitomycin C and *Bacillus* Calmette–Guérin vaccine in mice with orthotopic bladder tumors [8].

Taken together, these studies mentioned above support the notion that GZFL is a potential drug for bladder cancer by using intravesical therapy.

### 4.2. Ovarian Cancer

Ovarian cancer is a common malignant tumor for women aged >40 years. Radical surgery and chemotherapy are standard treatments for ovarian cancer [61]. However, resistance to chemotherapy agents has greatly restricted their use. Obviously, chemoresistant metastasis hinders survival and is a major cause of death [62].

GZFL has been used to treat ovarian cancer for more than 20 years in the clinic, which could increase chemotherapy efficacy, minimize side effects, and reduce chemoresistance. Explicitly, the microarray analyses have shown that GZFL treatment could deter the cell cycle, invasion, and migration-related genes in ovarian cancer cell lines SKOV3 by inhibiting protein kinase B (AKT)/glycogen synthase kinase 3 *β* (GSK3*β*) signaling pathway. Meanwhile, GZFL also reduced tumor growth/metastasis to the lung in xenograft mice [63]. In addition, one study reported that GZFL had a therapeutic potential against cisplatin-resistant ovarian cancers *in vitro* and *in vivo* by suppressing the expression level and function of permeability glycoprotein (P-gp) through blockage of the PI3K/AKT/mTOR pathway. Furthermore, the inhibitory effect of GZFL on tumor growth has been found in cisplatin resistance in human ovarian cancer cell line SKOV3/DDP xenograft nude mice [64]. What's more, serum derived from rats administrated with GZFL extract in cisplatin-resistant human ovarian cancer SKOV3/DDP cells was a promising way to overcome cisplatin-resistant by inhibiting the expression of metadherin (MTDH), inducing the expression of phosphatase and tensin homolog (PTEN), and improving the interaction between MTDH and PTEN [65].

The article "The Multiple Pharmacologic Functions and Mechanisms of Action of Guizhi Fuling Formulation" was published in 2022. Journal: Evid Based Complement Alternat Med.

### 4.3. Cervical Cancer

Cervical cancer is the primary cause of death among all gynecologic cancers. The imbalance of expression of matrix metalloproteinases (MMPs) and tissue inhibitors of metalloproteinases (TIMPs) can result in degradation of the extracellular matrix (ECM), which is a pivotal stage in tumor invasion [66]. One study reported that GZFL might restore the balance of MMPs/TIMPs and inhibit ECM degradation by decreasing MMPs activities and increasing TIMPs activities in HeLa cells which, eventually, interfered with the growth and invasion of cervical cancer cells *in vitro* and *in vivo* [67].

### 4.4. Breast Cancer

Breast cancer is one of the women's most common cancer, and there is an upward trend in the incidence. An experimental study found that the active pharmaceutical ingredient and its fraction from the GZFL capsule had a strong potential to deter the proliferation of human breast cancer MCF-7 cells and MDA-MB-231 cells in different doses and suppress the rate of cell growth in human umbilical vein endothelial cells (HUVECs) proliferation without toxicity [68]. In addition, the other study found that GZFL culture suppressed the proliferation of MCF-7 cells in the S phase by reducing the expression of CyclinA2, Cdk2, and EGFR [69]. In addition, GZFL exhibited the antiproliferation, proapoptosis, and antiangiogenesis activities in MDA-MB-231 cells mainly through inhibiting the PI3K and the mitogen-activated protein kinase (MAPK) signaling pathways [70].

### 4.5. Malignant Melanoma

Melanoma is an aggressive cutaneous cancer with a poor prognosis and high mortality. Meanwhile, cutaneous melanoma is the most prevalent type. Accumulating evidence reported that long noncoding RNAs (lncRNAs) highly expressed in malignant melanoma cells could promote cellular proliferation, migration, and invasion [71, 72].

The article "The Multiple Pharmacologic Functions and Mechanisms of Action of Guizhi Fuling Formulation" was published in 2022. Journal: Evid Based Complement Alternat Med.

One of those abnormal lncRNAs, TPT1-AS1, can target and bind to miR-671-5p and negatively regulate its level. However, miR-671-5p played a key role in suppressing osteosarcoma cell proliferation by blocking the cell cycle [73]. One study reported that GZFL might suppress the proliferation, migration, and invasion of human cutaneous malignant melanoma cells through the regulation of the TPT1-AS1/miR-671-5p molecular pathway [74].

## 5. Blood and Vascular Disease

Consolidated evidence indicates that GZFL has various effects on blood stasis by reducing blood viscosity and platelet aggregation, increasing blood flow rate and erythrocyte deformability, as well as dilation of arteries [75]. Patients suffering varicose veins in the legs often complain of subjective symptoms (malaise, numbness, coldness, pain, and pruritus) that lower their quality of life. One clinical study reported that GZFL relieved “oketsu” (impaired microcirculation, blood congestion) and skin perfusion pressure in patients with varicose veins in the legs [75].

The symptoms of sensory sequelae after a stroke are usually cold sensations and numbness, which result from an unregulated vasomotor system and low peripheral blood flow [76]. A clinical investigation using a visual analog scale (VAS) found that GZFL alleviated cold sensations and numbness in 22 stroke patients by improving the skin perfusion temperature through an increase in peripheral blood flow [77].

In addition, GZFL had improving effects on articular symptoms and endothelial dysfunction in rheumatoid arthritis (RA) patients by reducing plasma levels of soluble vascular cell adhesion molecule-1 (sVCAM)-1 and lipid peroxide (LPO) [78]. A clinical trial demonstrated that GZFL significantly increased the mean value of the natural logarithmic-scaled reactive hyperemia index (LRHI) and decreased levels of nonesterified fatty acid (NEFA), malondialdehyde, and sVCAM-1 in serum, which contribute to GZFL's beneficial effects on endothelial function in metabolic syndrome patients [79].

A study using live imaging techniques showed that GZFL possessed an antioketsu effect on microcirculation in murine subcutaneous vessels, including amelioration of arterioles vasodilation and erythrocyte congestion, increasing blood velocity in the subcutaneous capillary. Furthermore, the authors found that the effect of GZFL on improving oketsu was related to an increase in NO levels in the mesenteric arterial endothelium of rats [80]. In addition, impaired microcirculation can be caused by other factors, such as platelets/leukocytes aggregation on endothelial cells. A study using screen filtration pressure showed that GZFL and its main constituent (Moutan Cortex and Cinnamomi Ramulus) were associated with the inhibitory effects on collagen-induced platelet aggregation and impaired microcirculation in whole blood samples from guinea pigs [81].

The article "The Multiple Pharmacologic Functions and Mechanisms of Action of Guizhi Fuling Formulation" was published in 2022. Journal: Evid Based Complement Alternat Med.

High cholesterol concentrations in serum have key roles in the progression of hypercholesterolemia and nonalcoholic fatty liver disease (NAFLD), which are critical risk factors for many cardiovascular diseases, including atherosclerosis, hypertension, and myocardial infarction [82]. One study reported that GZFL improved atherosclerosis by downregulating the levels of triglyceride (TG), alkaline phosphatase (ALP), alanine aminotransferase (ALT), and ICAM-1 (a marker of activation of the endothelial cell) in the serum, as well ICAM-1 expression in the aorta, of rats fed a high-cholesterol diet [83]. Analysis of network pharmacology and molecular docking confirmed that AKT1, caspase-3 (CASP3), MAPK1, MAPK3, NOS2, and prostaglandin-endoperoxide synthase 2 (PTGS2) were GZFL's potential target genes against atherosclerosis [84]. Besides, GZFL alleviated Coronary Heart Disease (CHD) syndromes (such as elevated ST segment, increased levels of serum creatine kinase-MB (CK-MB) and lactic dehydrogenase (LDH), abnormal histopathological features) and downregulated TNF-*α* and IL-6 levels in acute myocardial ischemia (AMI) rats induced with isoproterenol [85].

Therefore, GZFL shows the potential for inhibiting the development of blood stagnation, vascular endothelial dysfunction, and atheromatous plaque by exerting antioxidative, anti-inflammatory, and immunoregulatory effects against many blood and vascular diseases.

## 6. Renal Failure

Chronic renal failure is the most common complication of diabetes mellitus. Furthermore, in recent years, increasing numbers of patients suffering from diabetic nephropathy have required dialysis therapy, which lead to a rise in the cost of cure [86].

Notably, traditional herbal medicines are considered to be an effective alternative medicine for diabetic nephropathy. One study in spontaneously diabetic WBN/Kob rats reported that GZFL obviously reduced urinary excretion of proteins and serum levels of creatinine, inhibited oxidative stress by decreasing 8-Hydroxy-deoxyguanosine (8-OHdG) release in urine and kidneys and hepatic lipid peroxidation, and showed protective effects on renal function by suppressing transforming growth factor *β*_1_ (TGF-*β*_1_)-induced fibronectin release in the renal cortex [87]. Similarly, GZFL has been exhibited to significantly reduce the levels of blood urea nitrogen and urinary excretion of proteins and mRNA expressions of osteopontin, TGF-*β*1, and fibronectin in the remnant kidney of nephrectomized rats. Thus, these studies suggest that GZFL can help to retard the aggravation of chronic renal failure [88].

The article "The Multiple Pharmacologic Functions and Mechanisms of Action of Guizhi Fuling Formulation" was published in 2022. Journal: Evid Based Complement Alternat Med.

Recently, several studies have indicated that solute carrier organic anion transporters (OATs), as membrane proteins, regulate the reabsorption and excretion of renal metabolic substrates and toxins, which are considered to be novel drug targets for nephrotoxicity [89]. Furthermore, the pharmacologic effects of GZFL on the functions of renal transporters have been investigated. GZFL can suppress the substrate-uptake activities of urate transporter 1 (URAT1), OAT1, and OAT3 in *Xenopus oocytes* and HEK293 human kidney embryonic cells [90]. Therefore, GZFL has been seriously considered to be a nephroprotective agent.

## 7. Inflammation

Accumulating studies have presented experimental evidence of GZFL for the treatment of inflammation. An abnormal immune reaction can trigger chronic inflammation in skin diseases such as psoriasis, chronic pigmented purpura, and atopic dermatitis. Thus, regulation of immune homeostasis and inflammation in the skin may be an efficacious therapeutic approach against skin disease [91].

A study reported that GZFL treatment alleviated the disease severity using clinical assessments (SCORAD index and VAS score) in patients with atopic dermatitis, particularly those presenting with chronic lichenification. Conversely, the level of serum lactate dehydrogenase (LDH) was also decreased significantly in atopic dermatitis patients after GZFL treatment according to laboratory assessments [92]. Studies have shown that GZFL treatment significantly suppressed levels of migration inhibitory factor (MIF, an initiator of proinflammatory cytokines) [93] and subsequent production of IL-6, IL-8, TNF-*α*, COX-2, and inducible nitric oxide synthase (iNOS) in lipopolysaccharide- (LPS-) stimulated cultured human dermal microvascular endothelial cells (HDMECs). These results imply that GZLF exhibited a potential for improving microvascular inflammation-mediated shin disease, such as chronic pigmented purpura [7]. In addition, GZFL extract significantly reduced levels of chemokine (macrophages are derived from chemokines (MDC), regulated upon activation of normal T cell expressed sequence (RANTES)), and production of IL-8 and IL-8 mRNA in TNF-*α*/interferon-gamma- (IFN-*γ*-) stimulated HaCaT human keratinocytes by blocking the signal transducer and activator of transcription 1 (STAT1) pathway, which contributed to the anti-inflammatory effect of GZFL on skin disorders [94]. Taken together, those data suggest that GZFL is a potent therapeutic drug for inflammation-associated skin diseases.

The article "The Multiple Pharmacologic Functions and Mechanisms of Action of Guizhi Fuling Formulation" was published in 2022. Journal: Evid Based Complement Alternat Med.

In addition, GZFL and its active complex can inhibit the inflammatory response by decreasing the secretion of IL-1*β*, TNF-*α*, and PGE2 in LPS-induced RAW264.7 cells [95]. Furthermore, proinflammatory chemokines factors contribute to the development of atherosclerosis and NAFLD. GZFL can downregulate the expression of MCP-1 and its receptor CC chemokine receptor 2 (CCR2) in the liver and adipose tissue to improve atherosclerosis in rats fed a high-cholesterol diet [83]. Furthermore, another study on neuroinflammation reported that GZFL also decreased levels of proinflammatory factors, such as NO, IL-1*β*, TNF-*α*, iNOS, COX-2, macrophage inhibitory protein- (MIP-) 1*α*, MCP-1, and IFN-*γ* inducible protein- (IP-) 10, RANTES, in LPS-stimulated BV2 microglia by blocking nuclear factor-kappa B (NF-*κ*B), extracellular signal-regulated kinase (Erk), c-Jun N-terminal kinase (JNK), and PI3K/AKT pathways. On the contrary, GZFL could increase the expression of anti-inflammatory factors, including IL-10 and Heme oxygenase 1 (HO-1), in LPS-stimulated BV2 microglia through activation of nuclear factor-E2-related factor-2 (NRF2) and cyclic adenosine monophosphate-response element-binding protein (CREB) pathways, suggesting that GZFL exhibited an anti-inflammatory effect on microglia-related neuroinflammatory disorders [96].

## 8. Brain Injury

Disability and death are common outcomes of ischemic stroke and are characterized by the interruption of cerebral blood flow. The postischemic inflammatory response exacerbates neuronal damage and loss, leading to neurological dysfunction in patients suffering from ischemic stroke. However, efficacious treatment approaches against stroke are lacking.

In Asia, extensive experiences and clinical research have indicated that traditional herbal medicine has beneficial effects on postischemic rehabilitation in stroke patients [97]. Studies demonstrated that GZFL administration elicits significant protective effects against cerebral ischemia/reperfusion injury through decreasing infarct areas and water contents of brain tissue in stroke rats, which is attributed to the anti-inflammatory properties of GZFL. As expected, GZFL treatment not only obviously reduced the levels of TNF-*α* and IL-1*β* but also elevated IL-10 levels in serum and brain tissue of rats with cerebral ischemia/reperfusion injury [10].

Recently, diabetes mellitus has been reported to induce neuronal loss and cognitive deficits [98]. One study showed that GZFL treatment ameliorated memory impairment in streptozotocin- (STZ-) induced hyperglycemic mice. Moreover, GZFL significantly reduced the number of TUNEL^+^ cells and caspase-3^+^ cells in the cortex and hippocampus of STZ-induced hyperglycemic rats. Similarly, the increased protein levels of caspase-3 and reduced Bcl-2 were reversed in the cortex and hippocampus by GZFL treatment in STZ-induced hyperglycemic rats [99]. A depression-related study found that GZFL could reverse the decreased body weight and food intake in reserpine-induced depression mice. Furthermore, GZFL improved depressive-like behaviors by regulating immune/endocrine dysfunction in depression mice, as evidenced by a decrease in corticosterone levels in plasma and mRNA expressions of proinflammatory factors in the hippocampus after GZFL treatment through activation of the BDNF-CREB pathway [100].

The article "The Multiple Pharmacologic Functions and Mechanisms of Action of Guizhi Fuling Formulation" was published in 2022. Journal: Evid Based Complement Alternat Med.

In general, these results mentioned above suggest that GZFL treatment may be beneficial for patients with ischemia- or diabetes mellitus-induced brain injury and depression.

## 9. Other Therapeutic Effects

Other therapeutic effects of GZFL have been reported in clinical and experimental studies. After GZFL treatment, dietary-induced obese mice showed an obvious decrease in serum levels of leptin, liver levels of TG, and cholesterol. In addition, GZFL also reduced the adipocyte accumulation and steatosis in the liver of dietary-induced obese mice by suppressing expressive of lipid metabolism-associated genes such as peroxisome proliferator-activated receptor-*γ* (PPA*γ*) and sterol-regulated element-binding protein 1 (SERBP1) [101]. GZFL and its active components exhibited immunomodulatory effects by enhancing the expression of CD80 and CD86 in splenic lymphocytes and the CD25/CD69 ratio in splenic T lymphocytes, suggesting that the pharmacologic mechanism of GZFL is also involved in the regulation of lymphocyte activation [102].

## 10. Safety and Toxicity

Security and toxicity evaluations of traditional Chinese medicine have drawn concerns. Negative side effects or toxicity of GZFL have been observed in patients with the gynecologic disease [103]. GZFL was not found to cause detectable carcinogenic or genotoxic effects in other studies [104, 105]. GZFL has been assessed for efficacy and safety in the treatment of dysmenorrhea by the USA Food and Drug Administration [106, 107]. Gratifyingly, GZFL has been exhibited to be very safe and efficacious with little adverse reaction in other studies [6, 108].

## 11. Conclusion

In summary, this review suggests that GZFL displays promising therapeutic effects for many kinds of diseases, which have been beyond the scope of the original prescription for gynecologic diseases. Moreover, a large number of clinical and experimental researches demonstrated that GZFL also was used to treat cancer, blood and vascular disease, renal failure, inflammation, and brain injury. Possibly due to its diverse bioactive components and pharmacologic activities, GZFL could target multiple signaling pathways involved in various diseases, such as blood circulation, inflammatory and immune factors, proliferation, and apoptosis. The multiple pharmacologic effects and possible mechanisms of action of GZFL are summarized in Table 1. Notably, anti-inflammatory and immunomodulatory effects of GZFL play a central role in treating various diseases, indicating that GZFL possesses a potential for strengthening the body resistance to eliminate pathogenic factors and optimize the body function, which conform to the strategy of the overall treatment in traditional medicine. However, much of the actual data from *in vivo* and *in vitro* experiments have sufficiently demonstrated obvious potential for GZFL to improve certain diseases, including cancer, renal failure, and brain injury, which are difficult to extrapolate these data to the clinical experiments. Thus, in order to prove the potential of GZFL in patients, a large number of rigorous designed and well-controlled clinical researches are required, which relate to the cellular and animal data to supply a strong cause-and-effect for their therapeutic potentials against the above diseases. At present, its deeply molecular mechanisms underlying different pharmacodynamic effects are not fully understood. Accordingly, in the future, we should fully combine GZFL's physical and chemical properties and conduct a new innovative research mode “from bedside to bench to bedside” to examine the pharmacodynamic effects and underlying mechanisms of GZFL and thereby enlighten the development of Chinese classic herbal formulation.

The article "The Multiple Pharmacologic Functions and Mechanisms of Action of Guizhi Fuling Formulation" was published in 2022. Journal: Evid Based Complement Alternat Med.

## Figures and Tables

**Table 1:** Summary of pharmacologic effects and targets of Guizhi Fuling Formulation (GZFL).

Diseases		Pharmacological effects and targets	Patient/Model	Refs.
Gynecologic diseases	Primary and secondary dysmenorrhea	Improvement (to some degree) in >80% of patients	Patients	[29]
		Induces smooth blood flow	Patients	[4]
		Improves acne vulgaris	Patients	[12]
		Reduces lamina propria edema and COX-2 expression	Oxytocin-induced ICR mice	[31]
		Downregulates the mRNA expressions of COX-1 and COX-2	Human umbilical vein endothelial cells	[32]
		Decreases NO, PGF_2*α*_, Ca^2+^, COX-2, OTR in uterine tissue suppresses uterus contractions, restrains intracellular Ca^2+^	Oxytocin-induced ICR mice Oxytocin-induced uterine strips and myometrial cells	[33]
		Reduces writhing times, PGF_2a_/PGE_2_ ratio in plasma, urinary metabolic deviations	Oxytocin-induced rats	[34]
		Reduces writhing times, and the number of spiral arteries and inflammatory cells in uterine tissues; Increases PGE_2_/PGF_2*α*_, 6-Keto-PGF_1*α*_/TXB_2_ ratio in plasma	Estradiol benzoate- and oxytocin -induced rats	[35]
	Uterine fibroids	Reduces uterine size and fibroids volume	Patients	[3]
		Relieves pelvic pain and the uterine fibroid symptoms and reduces the uterine size and fibroids volume	Patients	[39]
		Suppresses proliferation and promotes apoptosis and increases TSC2, FOXO by regulating the 14-3-3*γ* signal pathway	Human uterine leiomyoma cells	[40]
		Inhibits uterine fibroids growth by modulating Med12-mediated wnt/*β*-catenin signaling pathway	Estradiol benzoate- and progesterone-induced SD rats Human uterine leiomyoma cells	[41]
		Ameliorates endometrial hyperplasia through promoting p62-Keap1-NRF2-mediated ferroptosis	Estradiol-induced endometrial hyperplasia mice	[42]
		Inhibits proliferation and induces apoptosis by multiple pathways	Network pharmacology	[9]
	Endometriosis	Improves pregnancy rate, and decreases the recurrence rate Reduces estradiol and progesterone in serum	Patients	[45]
		Decreases the ratio of Bcl-2/Bax, survivin Increases caspase-3 and caspase-9	Endometrial cells of rats	[44, 46]
		Increases the percentage of CD4^+^ T cells, activity of NK cell Decreases MCP-1 and ICAM-1	Endometriosis model in rats	[47]
	Climacteric syndrome	Improves vasomotor symptoms, melancholia	Patients	[51]
		Improves sleep disturbance, perspiration, and reduces blood pressure, heart rate	Patients	[52]
		Ameliorates hot flashes by regulating CGRP	Patients	[54]
		Decreases the frequency and severity of hot flashes	Patients	[2]
	Polycystic ovary syndrome	Improves insulin resistance via regulating intestinal flora to control inflammation	PCOS rats with insulin resistance	[58]
		Inhibits granulosa cell autophagy and promotes follicular development to attenuate ovulation disorder by restoring PI3K/AKT/mTOR pathway		[59]
*Cancer*	Bladder cancer	Interferes with cell cycle progression by activating CHK2 and P21	Human bladder cancer cells	[60]
		Activates ATM/CHK2 and ATM/P53 pathways	Mouse bladder cancer cells	[8]
		Inhibits tumor growth	Orthotopic bladder cancer mice	
	Ovarian cancer	Suppresses cell cycle, invasion, and migration-related genes by inhibiting the AKT/GSK3*β* pathway	HEY and SKOV3 cells	[63]
		Reduces tumor growth and metastasis	Xenograft mice	
		Decreases P-gp by blocking the PI3K/AKT/mTOR pathway	SKOV3 and SKOV3/DDP cells	[64]
		Inhibits tumor growth	SKOV3/DDP xenograft nude mice	
		Inhibits MTDH expression, induces PTEN expression, and improves the interaction between MTDH and PTEN	SKOV3 cells and its cisplatin-resistant SKOV3/DDP cells	[65]
	Cervical cancer	Restores the MMP-TIMP balance Suppresses degradation of the extracellular matrix	Human cervical cancer (HeLa) cells	[67]
		Interferes with tumor growth and invasion	HeLa human cervical cancer xenograft mice	
	Breast cancer	Inhibits the proliferation Suppresses cell growth rate	MCF-7 and MDA-mb-231 cells HUVECs	[68]
		Inhibits the proliferation by reducing the expression of CyclinA2, Cdk2, and EGFR	MCF-7 cell	[69]
		Inhibits proliferation, angiogenesis and promotes apoptosis by regulating the PI3K and the MAPK pathways	MDA-MB-231 cells	[70]
	Malignant melanoma	Inhibits the proliferation, migration, and invasion by regulating the molecular axis of LncRNA TPT1-AS1/mir-671-5p	Human cutaneous malignant melanoma cells A375	[74]
Blood and vascular disease	Varicose veins legs	Improves subjective symptoms, “oketsu”, and skin perfusion pressure	Patients	[75]
	Cold sensation and numbness after stroke	Increases peripheral blood flow	Stroke patients	[77]
	Rheumatoid arthritis	Reduces sVCAM-1 and LPO	Patients	[78]
	Metabolic syndrome	Increases LRHI Decreases NEFAs, sVCAM-1, and malondialdehyde	Patients	[79]
	Oketsu (ischemia)	Induces vasodilation, increases blood velocity Decreases endothelial NO production	Mice subcutaneous vessels and rat mesenteric arterioles	[80]
	Platelet aggregation	Improves impaired microcirculation	Whole blood of guinea pigs	[81]
	Atherosclerosis	Downregulates TG, ALP, ALT and ICAM-1	High-cholesterol-diet rats	[83]
	Coronary heart disease	Alleviates CHD syndromes and regulates inflammatory responses	Isoproterenol-induced AMI rats	[85]
Renal failure	Diabetic renal disease	Reduces urinary protein excretion and serum creatinine, 8-OHdG, lipid peroxidation, fibronectin, and TGF-*β*_1_	Spontaneously diabetic WBN/Kob rats	[87]
	Chronic renal failure	Reduces blood urea nitrogen and urinary protein excretion, as well as mRNA expressions of osteopontin, TGF-*β*1, and fibronectin	Nephrectomized rats	[88]
	Nephrotoxicity	Suppresses substrate-uptake activities of URAT1, OAT1, and OAT3	*Xenopus* oocytes and HEK293 cells	[90]
Inflammation-related diseases	Atopic dermatitis	Alleviates disease severity and reduces serum LDH	Patients	[92]
	Chronic pigmented purpura	Suppresses MIF, IL-6, IL-8, TNF-*α*, COX-2, and iNOS	LPS-stimulated HDMECs	[7]
	Inflammatory skin disorders	Reduces chemokine production and p-STAT1	TNF-*α* and IFN-*γ*-induced HaCaT cells	[94]
	Inflammatory response	Decreases IL-1*β*, TNF-*α* and PGE2	LPS-induced RAW264.7 cells	[95]
	Atherosclerosis	Downregulates MCP-1 and its receptor CCR2	High-cholesterol-diet rats	[83]
	Neuroinflammatory disorders	Decreases NO, IL-1*β*, TNF-*α*, iNOS, COX-2, MIP-1*α*, MCP-1, IP-10, RANTES, NF-*κ*B, erk, JNK, and PI3K/AKT Increases IL-10, HO-1, NRF2, and CREB	LPS-induced BV2 microglia	[96]
Brain injury	Cerebral ischemia/reperfusion injury	Decreases infarct area and water content of brain tissue Reduces TNF-*α*, IL-1*β* increases IL-10 in serum and brain tissue	Rats	[10]
	Hyperglycemia and diabetes mellitus	Improves memory deficits Decreases TUNEL^+^ cells and caspase-3^+^ cells Reduces caspase-3 Increases Bcl-2	STZ-induced hyperglycemic mice and rats	[99]
	Depression	Increases body weight and food intake Improves depressive-like behavior Reduces corticosterone in plasma Decreases IL-1*β*, IL-6, and TNF-*α* Increases BDNF and p-CREB in the hippocampus	Reserpine-induced mice	[100]
Other diseases	Obesity	Decreases leptin, TG, and cholesterol	SHR rats and the DIO mice	[101]
	Immune-related disease	Enhances CD80 and CD86 and CD25/CD69 ratio	Spleen T lymphocytes	[102]

The article "The Multiple Pharmacologic Functions and Mechanisms of Action of Guizhi Fuling Formulation" was published in 2022. Journal: Evid Based Complement Alternat Med.

## Data Availability

The data are included in the article as table.
